The article "Antiproliferative and pro-apoptotic activity of melatonin analogues on melanoma and breast cancer cells" was retracted in 2025. Reasons: duplicated images; concerns about the images.

# Antiproliferative and pro-apoptotic activity of melatonin analogues on melanoma and breast cancer cells

**DOI:** 10.18632/oncotarget.20124

**Published:** 2017-08-10

**Authors:** Giuliana Gatti, Valeria Lucini, Silvana Dugnani, Angela Calastretti, Gilberto Spadoni, Annalida Bedini, Silvia Rivara, Marco Mor, Gianfranco Canti, Francesco Scaglione, Annamaria Bevilacqua

**Affiliations:** ^1^ Department of Medical Biotechnology and Translational Medicine, Università degli Studi di Milano, Milan, Italy; ^2^ Department of Oncology and Hemato-oncology, Università degli Studi di Milano, Milan, Italy; ^3^ Department of Biomolecular Sciences, Università degli Studi di Urbino “Carlo Bo”, Urbino, Italy; ^4^ Department of Food and Drug, Università degli Studi di Parma, Parma, Italy

**Keywords:** melatonin analogues, melatonin receptors, anti-cancer drugs, melanoma, breast cancer

## Abstract

Melatonin plays different physiological functions ranging from the regulation of circadian rhythms to tumor inhibition, owing to its antioxidant, immunomodulatory and anti-aging properties. Due to its pleiotropic functions, melatonin has been shown to elicit cytoprotective processes in normal cells and trigger pro-apoptotic signals in cancer cells. The therapeutic potential of melatonin analogues prompted us to investigate the *in vitro* and *in vivo* antitumor activity of new melatonin derivatives and explore the underlying molecular mechanisms. The experiments revealed that the new melatonin analogues inhibited the growth of melanoma and breast cancer cells in a dose- and time-dependent manner. In addition, our results indicated that melatonin derivative UCM 1037 could induce apoptosis in melanoma and breast cancer cells, as well as cell necrosis, in MCF-7. Together, apoptosis and necrosis could be two possible mechanisms to explain the cytotoxic effect of the melatonin analogue against cancer cells. The suppression of tumor growth by the melatonin analogues was further demonstrated *in vivo* in a xenograft mice model. A decrease in the activation of MAPK pathway was observed in all cancer cells following UCM 1037 treatment. Overall, this study describes a promising antitumor compound showing antiproliferative and cytotoxic activity in melanoma and breast cancer cells.

## INTRODUCTION

The N-acetyl-5-methoxytryptamine, or melatonin, is an indolic hormone mainly synthesized and secreted by the pineal gland from the essential amino acid tryptophan [1]. In addition, there is also evidence for melatonin production in other organs, including the retina, gastrointestinal tract, skin, bone marrow, and immune system cells [2]. Melatonin production is regulated by photoperiod as its synthesis and secretion are repressed by light and induced in response to darkness [3].

Melatonin plays pleiotropic roles in maintaining health and preventing disease [4]. A plethora of pathological disorders have been associated with the reduction of circulating melatonin levels, including aging, metabolic syndrome, type 2 diabetes, immune diseases, hypertension, mood and cognitive disorders, and cancer [5–8].

Over the last decades, significant research efforts have been devoted to defining the role of melatonin in the pathogenesis of cancer and its possible therapeutic application. It has been shown that melatonin, under both *in vitro* and *in vivo* conditions, inhibits the growth of some cancer cells [9–11], although its role and mechanism of action are still controversial. Besides its antiproliferative role in cancer cells, melatonin can also exert cell protection functions, acting as a scavenger for reactive oxygen and reactive nitrogen species and activating cytoprotective enzymes [12–14].

Melatonin can exert its multiple actions by various receptor-dependent and receptor-independent mechanisms [15]. Accordingly, melatonin interacts with different cellular components, including intracellular proteins, nuclear membrane receptors, and cell membrane receptors. Two membrane receptors, MT_1_ (formerly called Mel1a or ML1A) and MT_2_ (formerly called Mel1b or ML1B) were cloned [16, 17] and pharmacologically characterized [18]. They are both members of the superfamily of G-protein coupled receptors, traditionally considered to function as monomers, but they can also act as homodimers and heterodimers. When they act as monomers, the receptor signaling inhibits protein kinase A (PKA) pathway and CREB phosphorylation. The MT_1_ receptor also modulates phosphorylation of mitogen-activated protein kinase 1/2 (MAPK1/2) and extracellular signal–regulated kinase 1/2 (ERK1/2) [19]. As homo and heterodimers human MT_1_ and MT_2_ receptors alter phospholipase C (PLC) and protein kinase C (PKC) pathways [20]. In addition, melatonin can cross cell membranes exerting several receptor-independent effects [21]. These include the activation of different cascades and/or ion channels resulting in cAMP decrease, PLC, PKC, MAP kinase and phosphatidylinositol 3 kinase (PI3K)/Akt pathways activation, Ca^2+^-activated K^+^ as well as voltage-gated Ca^2+^ channels modulation [22].

The effects of melatonin have been studied in numerous types of tumors, leading to the general conclusion that melatonin inhibits cell proliferation and induces apoptosis in most tumor cell lines and reduces tumor growth in cancer murine models. Moreover, melatonin suppresses tumor metastases by regulating cell adhesion, extracellular matrix remodeling, epithelial-mesenchymal transition, cytoskeleton reorganization and angiogenesis [11].

The effects of melatonin on different tumors are quite diverse, ranging from antioxidant, immune-modulatory and enzyme regulatory, to regulation of various kinases and transcription factors or via activation of its G-protein coupled MT_1_/MT_2_ receptors. Radiolabeled ligands and selective MT_1_ and MT_2_ melatonin receptor agonists and antagonists, are currently used as tools for studying melatonin functions and some receptor agonists have also been approved for clinical use, mainly to treat sleep disorders or major depression [23, 24].

Herein, we studied new synthetic indole melatonin analogues for their ability to inhibit proliferation and induce apoptosis in cancer cell lines and to reduce tumor growth in a cancer mouse model.

## RESULTS

### Human receptor binding characterization of the new melatonin derivatives

The new melatonin analogues (UCM 976, UCM 1032, UCM 1033, UCM 1037) were designed starting from previous indole melatonin receptor ligands replacing their 5-methoxy group with a moiety known to induce some MT_1_ selectivity such as the more lipophilic phenylbutoxy one (Table 1).

**Table 1:** Chemical structures of melatonin and of the new synthesized melatonin analogues

Compound	Structure	cLogP^a^
Melatonin		0.71
UCM 976		3.55
UCM 1032		4.26
UCM 1033		5.28
UCM 1037		4.26

^a^Calculated logP values (cLogP) were calculated using ChemBioDraw Ultra 14.0 (Cambridge Soft, Cambridge, MA, USA).

The melatonin derivatives were evaluated for their binding affinity and intrinsic activity at human MT_1_ and MT_2_ receptors stably transfected in NIH3T3 mouse fibroblasts and the results are reported in Table 2.

**Table 2:** Human melatonin receptor binding affinity and relative intrinsic activity of melatonin analogues

	MT_1_		MT_2_	
	pKi (± s.d.)	IAr (± s.d.)	pKi (± s.d.)	IAr (± s.d.)
Melatonin	9,623 ± 0,037	1,000 ± 0,001	9,66 ± 0,017	1,000 ± 0,001
UCM 976	8,46 ± 0,041	0,702 ± 0,06	7,30 ± 0,064	0,392 ± 0,022
UCM 1032	8,73 ± 0,131	0,942 ± 0,01	7,87 ± 0,106	0,759 ± 0,076
UCM 1033	8,62 ± 0,214	0,997 ± 0,003	7,73 ± 0,160	0,859 ± 0,015
UCM 1037	8,86 ± 0,148	0,930 ± 0,044	7,72 ± 0,140	0,776 ± 0,011

All the new compounds displayed affinity for MT_1_ receptor in the nanomolar range and modest selectivity (approximately 10-fold) with respect to MT_2_ receptor. In particular, MT_1_ and MT_2_ binding affinity measures for UCM 976 are comparable to those previously reported [25] for receptors expressed in CHO cells. Compared with the corresponding N-anilinoethylamide ligand [26], carrying the same phenylbutyloxy side chain, this indole derivative has a slightly lower MT_1_ selectivity. As expected from structure-activity relationships for indole receptor ligands, insertion of a lipophilic substituent in position 2 increases binding affinity at both receptor subtypes, as well as intrinsic activity. Indeed, functional assays showed full agonist behavior at both melatonin receptor subtypes, except UCM 976 which can be considered as a partial agonist at the MT_2_ receptor.

### Antiproliferative and cytotoxic effects of melatonin analogues on cancer cell lines

Melatonin has been shown to inhibit growth of a wide variety of cancer cells, including hormone-dependent and hormone-independent tumors. In this study, we chose to investigate the antiproliferative and cytotoxic activity of melatonin analogues in hormone-dependent (breast cancer) and hormone-independent (melanoma) cancer types. DX3 and WM-115 melanoma, as well as MCF-7 and MDA-MB231 breast cancer cells were first assessed for MT_1/2_ expression by Western blot analysis (Figure 1). MT_1/2_ receptors were detectable in all the cell lines examined. NIH3T3 mouse fibroblasts stably transfected with MT_1_ (NIH3T3-1A) and MT_2_ receptor (NIH3T3-1B) were used as positive controls for MT_1_ and MT_2_ respectively, wild type NIH3T3 cell lysate was loaded as a negative control.

**Figure 1:** MT_1/2_ receptors expression in different cell lines Western blot analysis showing the expression of MT_1/2_ receptors in NIH3T3, NIH3T3-1A, NIH3T3-1B, DX3, WM-115, MCF-7 and MDA-MB231 cells. The assay was performed on 30 μg of protein extract from each cell line. Tubulin is shown as a loading control.

The antiproliferative effects of the synthesized compounds were evaluated in the cancer cell lines by the XTT assay that detects the cellular metabolic activities. DX3, WM-115, MCF-7 and MDA-MB231 cells were seeded in 96-well plates and 24 hours later were treated with 0.1% dimethyl sulfoxide (DMSO) dissolved in cultured medium or with melatonin (10^−5^−10^−3^ M), UCM 976, UCM 1032, UCM 1033 and UCM 1037 (10^−6^−10^−4^ M) in 0.1% DMSO and cultured for 24, 48 and 72 hours. The XTT assay revealed that most compounds had an antiproliferative effect in a dose- and time-dependent manner (Figures 2 and 3). In particular, UCM 1033 and UCM 1037 10^−4^ M showed the maximum effect in DX3 cells reducing cell viability to 40% and 37% after 48 hours and to 25% and 22% after 72 hours respectively compared to DMSO treated cells (Figure 2B and 2C). The same melatonin analogues caused an even more marked decrease of cell proliferation in WM-115 cells, with UCM 1033 and UCM 1037 10^−4^ M reducing cell number to 21% and 23% after 48 hours and to 14% and 10% after 72 hours respectively compared to DMSO treated cells (Figure 2E and 2F). Melatonin did not inhibit significantly cell proliferation of melanoma cells at the same dose.

**Figure 2:** Cell viability of melanoma cells treated with different doses of melatonin analogues DX3 and WM-115 cells were seeded as described in Materials and Methods and treated with 0.1% DMSO, melatonin (MLT), UCM 976, UCM 1032, UCM 1033 and UCM 1037 dissolved in 0.1% DMSO at the indicated doses expressed in molarity (M). DX3 cell viability was evaluated by XTT assay after 24 (panel **A**), 48 (panel **B**) and 72 hours (panel **C**). Panels **D**–**F** show WM-115 cell viability evaluated as described above after 24, 48 and 72 hours respectively. Graphic bars represent percentage of living cells in each sample. The results have been normalized to 0.1% DMSO treated cells and are the means of three independent experiments ± s.d. *P-value < 0.001 *versus* 0.1% DMSO treated cells.

**Figure 3:** Cell viability of breast cancer cells treated with different doses of melatonin analogues MCF-7 and MDA-MB231 cells were seeded as described in Materials and Methods and treated with 0.1% DMSO, melatonin (MLT), UCM 976, UCM 1032, UCM 1033 and UCM 1037 dissolved in 0.1% DMSO at the indicated doses expressed in molarity (M). After 24 (panel **A**), 48 (panel **B**) and 72 hours (panel **C**) MCF-7 cell viability was evaluated by XTT assay. Panels **D**–**F** show MDA-MB231 cell viability evaluated as described above after 24, 48 and 72 hours respectively. Graphic bars represent percentage of living cells in each sample. The results have been normalized to 0.1% DMSO treated cells and are the means of three independent experiments ± s.d. *P-value < 0.001 *versus* 0.1% DMSO treated cells.

The effects of melatonin and its analogues on cell proliferation were also investigated on two human breast cancer cell lines (Figure 3). The XTT assay showed that all melatonin derivatives had an antiproliferative effect on MCF-7 cells in a dose- and time-dependent manner, although to different extents (Figure 3A–3C). In particular, UCM 1032 10^−4^ M showed the maximum effect reducing cell viability to 14% compared to DMSO treated cells after 72 hours. This difference was significant also *versus* melatonin 10^−3^ M. Similar results were obtained in MDA-MB231 cells (Figure 3D–3F). The reduction of cell viability estimated as the percentage relative to the mean of absorption obtained from the 0.1% DMSO treated cells after 72 hours was 37%, 14%, 26% and 31% for UCM 976, UCM 1032, UCM 1033 and UCM 1037 (10^−4^ M) respectively. Cell viability reduction was significant compared to both DMSO and melatonin (10^−3^ M) treated cells.

UCM 1037 was selected to assay its cytotoxicity in DX3, WM-115, MCF-7 and MDA-MB231 cells by Annexin-V and Propidium Iodide staining for apoptosis. Cells were seeded in Petri dishes and 24 hours later were treated with 0.1% dimethyl sulfoxide (DMSO) dissolved in cultured medium or with UCM 1037 (10^−4^ M) in 0.1% DMSO. After 24, 48 and 72 hours, cells were stained with Annexin-V/PI for the quantitative analysis of apoptotic and necrotic cells [27]. Cytofluorimetric analysis revealed that 88% of DX3 cells treated with UCM 1037 10^−4^ M were Annexin-positive/PI-positive after 72 hours of treatment (Figure 4A), implicating that the vast majority of UCM 1037 treated cells were in late apoptosis/secondary necrosis. WM-115 cells treated as described above exhibited a time-dependent cytotoxicity induced by UCM 1037 10^−4^ M, with 22%, 52% and 65% of Annexin-positive cells after 24, 48 and 72 hours respectively (Figure 4B). MCF-7 cells showed a different pattern of cytotoxicity induced by the melatonin analogue, with 80% of Annexin-negative and PI-positive cells after 72 hours, representative of necrotic death in MCF-7 cells treated with UCM 1037 (Figure 4C). MDA-MB231 cells subjected to the same treatments exhibited a time-dependent cytotoxicity induced by UCM 1037, with 18%, 38% and 44% of Annexin-positive cells after 24, 48 and 72 hours respectively (Figure 4D). Microscopic images of cells were also taken and are shown in Supplementary Data (Supplementary Figures 1 and 2).

**Figure 4:** Detection of apoptosis and necrosis by Annexin-V/Propidium Iodide assay DX3 (panel **A**), WM-115 (panel **B**), MCF-7 (panel **C**) and MDA-MB231 (panel **D**) cells were treated with 0.1% DMSO or with UCM 1037 10^−4^ M dissolved in 0.1% DMSO. After 24, 48 and 72 hours cells were simultaneously stained with Alexa Fluor-488-Annexin-V and Propidium Iodide and analyzed by flow cytometry to determine apoptosis and necrosis as described in Materials and Methods. One representative experiment out of three performed with similar results is shown in the cytograms. The white bars of the graphs below the cytograms represent the percentage of apoptotic cells (A+/PI−; A+/PI+), while the red bars represent the percentage of necrotic cells (A−/PI+) treated as described above.

### Oncostatic effect of melatonin analogues on a melanoma mouse model

The experiments described in the previous paragraph demonstrated that UCM 1033 and UCM 1037 melatonin analogues were the most effective compounds in suppressing cancer cell growth in melanoma cells. For this reason, DX3 cell line was chosen to perform *in vivo* experiments to test oncostatic effects of UCM 1033 and UCM 1037 on a human melanoma xenograft mouse model.

Data displayed in Figure 5 show that UCM 1033 melatonin analogue significantly inhibited melanoma tumor growth by 40%, while UCM 1037 inhibition of cancer growth reached 90% compared to vehicle treated mice. The same dose of melatonin did not induce significant tumor growth suppression.

**Figure 5:** Antitumor activity of melatonin analogues in a xenograft mouse model DX3 xenograft mice were injected s.c. with 5% DMSO (control), melatonin (MLT), UCM 1037, UCM 1033 16mg/kg in 5% DMSO every day for three weeks. All animals were then anesthetized and tumors removed and weighted. (**A**) Tumor xenografts from one of three independent experiments are shown. (**B**) Values of tumor mass are expressed as the mean ± s. d. (*n* = 3). *P < 0.001, compared with the control group.

### Antiproliferative effects of UCM 1037 in cell clones expressing MT_1_ and MT_2_ receptors

In order to address the hypothesis that UCM 1037 antiproliferative activity is, at least in part, mediated by melatonin receptors, NIH3T3 mouse fibroblasts, as well as NIH3T3-1A and NIH3T3-1B cell clones expressing MT_1_ and MT_2_ respectively, were treated with 0.1% DMSO dissolved in cultured medium or with 10^−4^ M UCM 1037 in 0.1% DMSO and cultured for 24, 48 and 72 hours. The XTT assay revealed that while wild type NIH3T3 cell proliferation was not significantly affected by UCM 1037, the melatonin analogue had an antiproliferative effect in a time-dependent manner on NIH3T3-1A and NIH3T3-1B cell clones (Figure 6A). This decrease in cell proliferation was not due to cell death since cell viability was greater than 92% in both NIH3T3 clones following 72 hours of treatment (Figure 6B).

**Figure 6:** Cell viability of NIH3T3 cells treated with UCM 1037 NIH3T3, NIH3T3-1A and NIH3T3-1B cells were treated with 0.1% DMSO or with UCM 1037 10^−4^ M dissolved in 0.1% DMSO. After 24, 48 and 72 hours cell viability was evaluated by XTT assay (**A**) and Trypan blue dye exclusion assay (**B**). In panel A bar graph represents the percentages of living cells normalized to 0.1% DMSO treated cells. In panel B bar graph represents the percentage of dead cells in each sample. Data are the means of three independent experiments ± s.d. *P-value < 0.001 *versus* 0.1% DMSO treated cells.

### Effects of UCM 1037 on protein expression

The correlation between the occurrence of cell death and the changes in the expression levels of different proteins involved in apoptosis and in MT_1/2_ mediated response induced by UCM 1037 was next investigated. Specifically, MAPK and Akt signaling pathways have been chosen for their key roles in the antiproliferative effects of melatonin [28–30]. The expression of molecules regulating the apoptotic pathway, such as Bcl-2, Bax and caspase 3 has also been analyzed.

A short term time course was performed in DX3, WM-115, MCF-7 and MDA-MB231 cells treated with DMSO 0, 1% or UCM 1037 10^−4^ M. Western blot analysis showed that phosphorylated Akt at serine 473 (p-Akt) increased by 80% in DX3 cells treated with UCM 1037 compared to DMSO control, while p-MAPK levels decreased up to 50% upon UCM 1037 treatment (Figure 7A). Western blot analysis in WM-115 melanoma cells confirmed that UCM 1037 significantly inhibited phosphorylation of MAPK (up to 30% compared to DMSO treated cells) but not Akt (Figure 7B). The expression of MAPK and Akt was not altered by UCM 1037 in both melanoma cell lines.

**Figure 7:** Time course of protein expression in UCM 1037 melanoma treated cells DX3 (panel **A**) and WM-115 (panel **B**) cells were treated with DMSO 0.1% or UCM 1037 10^−4^ M for 0, 10, 30, 60, 120, 240 minutes and then subjected to Western blot analysis. Blots are shown for p-Akt, Akt, p-MAPK, MAPK, Bcl-2, caspase-3, Bax proteins with their corresponding tubulin controls. The black triangle points to the cleaved caspase-3 form. One representative blot is shown of three independent experiments. Bar charts show quantification of p-Akt, p-MAPK, Bcl-2, and Bax protein levels in DMSO (white bars) and UCM 1037 (black bars) treated cells. Densitometric data were normalized *versus* tubulin and results are presented as relative percentage of protein levels at 0 hours. Each bar represents the mean ± s.d. of three independent experiments.

Next, we detected the expression of the pro-apoptotic proteins caspase-3 and Bax, as well as the anti-apoptotic protein Bcl-2. Treatment with UCM 1037 effectively induced caspase-3 cleavage in DX3 cells (Figure 7A), but not in WM-115 cells (Figure 7B). In contrast, Bcl-2 expression did not change in DX3 cells, while it decreased by 65% in WM-115 cells after one hour of treatment with UCM 1037. No changes in Bax levels were observed in both cell lines.

To further confirm that the Akt and MAPK signaling pathways are involved in the UCM 1037 mediated inhibition of proliferation in breast cancer cells, the phosphorylated forms of the above mentioned proteins were analyzed in MCF-7 (Figure 8A) and MDA-MB231 cells (Figure 8B). Western blot analysis revealed that in both breast cancer cell lines p-Akt decreased dramatically upon treatment with UCM 1037, up to 20% and 10% in MCF-7 and MDA-MB231 respectively. Similarly, p-MAPK levels fast decreased after treatment with UCM 1037. Bcl-2 expression did not change in both breast cancer cells, while cleaved caspase-3 strongly increased only in MDA-MB231 cells upon treatment with UCM 1037. Bax levels did not change after UCM 1037 treatment in both breast cancer cell lines.

**Figure 8:** Time course of protein expression in UCM 1037 breast cancer treated cells MCF-7 (panel **A**) and MDA-MB231 cells (panel **B**) cells were treated with DMSO 0.1% or UCM 1037 10^−4^ M for 0, 10, 30, 60, 120, 240 minutes and then subjected to Western blot analysis. Blots are shown for p-Akt, Akt, p-MAPK, MAPK, Bcl-2, caspase-3, Bax proteins with their corresponding tubulin controls. The black triangle points to the cleaved caspase-3 form. One representative blot is shown of three independent experiments. Bar charts show quantification of p-Akt, p-MAPK, Bcl-2, and Bax protein levels in DMSO (white bars) and UCM 1037 (black bars) treated cells. Densitometric data were normalized *versus* tubulin and results are presented as relative percentage of protein levels at 0 hours. Each bar represents the mean ± s.d. of three independent experiments.

## DISCUSSION

Melatonin is a key element of the homeostatic mechanisms of the organism and it is involved in regulating a large number of physiological processes. Based on the plethora of biological roles played by melatonin, we can expect to find, among its analogues, potential drugs for treatment of metabolic and endocrine disorders as well as oncological diseases. Accordingly, melatonin receptors have emerged as appealing therapeutic targets for anticancer therapies over a wide range of cancer types [24]. Indeed, in the past decades several molecules which specifically bind to melatonin receptors have been tested for their role in the prevention or treatment of pathological conditions [31–33].

In this study, four indole melatonin analogues were synthesized and their antiproliferative and pro-apoptotic effects were analyzed in melanoma and breast cancer cell lines. According to the results of the cell viability assays, all the tested compounds (10^−4^ M) showed significant antiproliferative effects in all cell lines after 72 hours of treatment, even if only UCM 1037 demonstrated significant antiproliferative effect at the 10^−6^ M concentration in DX3, MCF-7 and MDA-MB231 cells. In breast cancer cell lines, UCM 1037 significantly inhibited cell viability in a time-dependent manner, although to a lesser extent than in DX3 cells. MCF-7 and MDA-MB231 cells displayed maximum inhibition of cell proliferation upon UCM 1032 treatment, but this melatonin analogue failed to significantly reduce cell number at the 10^−6^ M concentration. As previously reported [9, 10, 30, 34], millimolar concentrations of melatonin inhibited cancer cell viability, while lower concentrations had no effect on cancer cell proliferation. While melatonin has the highest binding affinity for its MT_1_ and MT_2_ receptors, it showed no or minimal antiproliferative activity. On the contrary, all melatonin derivatives caused a reduction of cell viability at various extents in the different cancer cell lines examined. This discrepancy between antiproliferative activity and affinity at melatonin receptors could arise from different reasons. First, melatonin has a range of known effects, either receptor-mediated or not, which protect cells form different damaging factors [35]. Thus, the cytostatic activity of melatonin derivatives could just emerge as the result of MT_1/2_ mediated antiproliferative effects and the lack of melatonin non-receptor mediated cytoprotective effects. On the other hand, activity on DX3 and WM-115 melanoma cells was significantly higher for compounds having a substituent (halogen or phenyl) at the position 2 of the indole nucleus and paralleled the increase in compound lipophilicity. Thus, while antiproliferative activity may be attributed to the receptor-mediated actions of these compounds, the hypothesis that it may be modulated by compound ability to interact with lipophilic compartments of the cells and/or be due to some, yet uncharacterized, off target cannot be ruled out. Melatonin has been previously shown to have oncostatic effects on melanoma *in vitro* and *in vivo* [36–37], yet melanoma cells proliferation can be differentially suppressed by melatonin upon different conditions, such as synchronized *versus* unsynchronized growth, cell lineage, melatonin receptor-dependent and independent mechanisms [36, 38].

Since the cytotoxic effect of melatonin seems to occur only in specific types of tumors and is not as widespread as its oncostatic action [9], we tested the hypothesis that UCM 1037 could exert a pro-apoptotic activity on cancer cell lines. The flow cytometric analysis after Annexin-V/PI staining confirmed the cytotoxic activity of UCM 1037 on DX3, WM-115, MCF-7 and MDA-MB231 cells, although the cell death mechanisms activated by the melatonin analogue were different in the cell lines that we considered. In particular, UCM 1037 exhibited a pro-apoptotic activity in melanoma cells as well as in MDA-MB231 breast cancer cells, while it induced mostly necrosis in MCF-7 cells. Overall our results indicated that UCM 1037 may induce different cell death pathways to wield its cytotoxic effect in diverse cancer cells.

We next investigated the anti-tumor activity of UCM 1033 and UCM 1037 (16 mg/Kg) *in vivo* and we revealed that melatonin analogues suppressed tumor growth of DX3 melanoma cells xenograft mice model to a much greater extent than melatonin administered at the same dose. The antiproliferative effect of UCM 1037 was higher than that of UCM 1033, while the two compounds did not substantially differ in the *in vitro* cell viability tests on DX3 cells. This may be due to differences in lipophilicity, which may result in differential tissue distribution. However, the possibility that the two compounds may bind an off target with different affinities, and that this putative off target has different relevance in the *in vitro* and *in vivo* experiments, respectively, cannot be ruled out. Overall our findings point out the antiproliferative and pro-apoptotic properties of the newly synthetized melatonin analogue both *in vitro* and *in vivo*.

These findings prompted us to further investigate the effects of UCM 1037 in the signaling pathways involved in antiproliferative and pro-apoptotic actions of the melatonin derivative. Since both MT_1_ and MT_2_ are implicated in controlling cellular growth in response to melatonin, we evaluated UCM 1037 antiproliferative effects in NIH3T3-1A and NIH3T3-1B clones compared to wild type NIH3T3 fibroblasts (Figure 6). Cell viability assays revealed that both clones displayed a significant inhibition of cell proliferation compared to NIH3T3 cells, indicating that the antiproliferative activity of the melatonin analogue is receptor-dependent. Moreover, these experiment also demonstrated that UCM 1037 10^−4^M is not cytotoxic in normal cells, since cell viability was not affected in NIH3T3 treated clones.

As previously stated, due to the lipophilic nature of UCM 1037 (Table 1), receptor-independent effects could also be envisaged, with multiple signaling leading to modulation of different cascades. Several studies using different cell types indicated that MAPK and Akt signaling pathways are associated with melatonin-mediated antiproliferative actions [28–30]. We highlighted that the melatonin analogue can trigger and/or inhibit these pathways differently in the cell lines examined. According to our data, UCM 1037 inhibits MAPK phosphorylation in all cell lines, although to different extents. MAPK/ERK pathway is known to be modulated by melatonin receptors and melatonin antiproliferative and anti-metastatic activities have been proved to involve multiple pathways including inhibition of p38 MAPK [30, 39]. Our results suggest that the inhibition of MAPK phosphorylation following UCM 1037 administration is indeed triggered by the melatonin analogue and this action might be mediated by the melatonin receptors, which are expressed in the cell lines examined (Figure 1).

The Akt pathway was affected quite differently in the diverse cell lines: p-Akt increased in DX3 cells, remained unaffected in WM-115 cells, while it dramatically decreased in breast cancer cell lines. Actually, melatonin was previously shown to inhibit Akt phosphorylation in MCF-7 [29] and MDA-MB231 cells [28]; though it was recently observed that melatonin could upregulate the PI3K/Akt pathway in other model systems [40, 41], including a melanoma cell line [42].

The mechanisms of melatonin-dependent cell death in cancer are still controversial and data presented in this paper confirm some of the discrepancies observed by others [43]. In fact, although an increase in the apoptotic fraction of cells was induced by UCM 1037 in DX3, WM-115 and, to a lesser extent, in MDA-MB231 cells, no effects were visible on Bax levels up to 72 hours after the compound administration (Figures 7, 8 and data not shown). In contrast, cleaved forms of caspase-3 were detected in DX3 and MDA-MB231 cells after one hour, indicating that UCM 1037 induces apoptosis by activating a caspase cascade in these cell lines. Caspase-3 was not cleaved in WM-115 cells, but the anti-apoptotic Bcl-2 protein expression was inhibited following UCM 1037 treatment. However, no changes in Bcl-2 protein levels were observed in the other cell lines. These results contrast with the findings of other studies showing that melatonin modulates Bcl-2/Bax balance in cancer cells [44–47].

A different mechanism must be envisaged for MCF-7 cells, where the expression of caspase-3 is still controversial. We and others [48] were able to detect the uncleaved form of this caspase in Western blots, but most studies report that MCF-7 do not express caspase-3. It has been demonstrated that even caspase-3-deficient MCF-7 cells can undergo apoptosis following a variety of stimuli [49], nevertheless Annexin V/PI staining demonstrated that UCM 1037 is able to induce necrosis in the MCF-7 cells. For this reason we suggest that apoptosis and necrosis could be two possible mechanisms to explain the growth-inhibition of melatonin analogue against cancer cells.

These results highlight that UCM 1037 mode of action is cell line dependent and the differences in cell types could underlie the lack of an apparent change in the apoptotic proteins in most cell lines as well as the different cell death processes observed. Since melatonin has the ability to exert its effects with or without a receptor and modulates many different pathways, melatonin analogue's mechanisms are difficult to interpret and a complete understanding of how UCM 1037 exerts its antiproliferative and cytotoxic effects is still not well defined.

Furthermore, pro-apoptotic effects of melatonin derivatives can be counter-intuitive, since high concentrations of melatonin have been shown to inhibit cell death and to protect normal cells against oxidative damage. However, we have observed that melatonin analogues can trigger cell death, both in cultured cancer cells and *in vivo*, suggesting that these molecules could enhance the effect of chemotherapeutic drugs.

In conclusion, novel melatonin analogues described in this paper demonstrated to be antiproliferative compounds with significant cytotoxic activity in melanoma and breast cancer cells. The anticancer effects of melatonin in many tumor cells have attracted considerable attention and the number of related studies is rapidly increasing [50]. The development of the new melatoninergic ligands which could be used both for scientific research and in medical practice is raising alongside [20]. The study of synergistic relationships between melatonin analogues and anti-cancer drugs is a promising field, and these compounds could significantly strengthen the cytostatic and the cytotoxic effects triggered by conventional antineoplastic drugs.

## MATERIALS AND METHODS

### Melatonin analogues synthesis

The new melatonin analogues were prepared by *O*-alkylation of *N*-acetyl-5-hydroxytryptamine with 1-bromo-4-phenylbutane in the presence of sodium hydride (UCM 976) and subsequent C2-indole halogenation with phenyltrimethylammonium tribromide (UCM 1032) or with iodine and silver triflate (UCM 1037). The 2-phenyl melatonin analogue (UCM 1033) was prepared from *O*-demethyl-2-phenylmelatonin (previoulsy obtained by ether cleavage of 2-phenylmelatonin using boron tribromide) and 1-bromo-4-phenylbutane in the presence of sodium hydride.

The experimental synthetic procedures used to prepare the new melatonin analogues and their characterization are available as Supplementary Data.

### Human melatonin receptors binding assay

The two radioligands, 2-[^125^I]iodomelatonin (specific activity, 2000 Ci mmol^−1^) and [^35^S]GTPγS ([^35^S]guanosine-5′-O-(3-thio-triphosphate), specific activity 1000 Ci mmol^−1^, were purchased from PerkinElmer. Binding affinities were determined using 2-[^125^I]iodomelatonin as the labeled ligand in competition experiments on cloned human MT_1_ and MT_2_ receptors expressed in NIH3T3 mouse fibroblast cells [51–53]. Cell membranes were incubated for 90 min at 37°C in binding buffer (Tris-HCl, 50 mM, pH 7.4). The final membrane concentration was 5–10 μg of protein per tube. The membrane protein level was determined in accordance with a previously reported method [54]. 2-[^125^I] Iodomelatonin (100 pM) and different concentrations of melatonin (10^−10^−10^−6^ M) or of the melatonin analogues were incubated with the receptor preparation for 90 min at 37°C. Nonspecific binding was assessed with 10 μM melatonin; IC_50_ values were determined by nonlinear fitting strategies with the program PRISM (GraphPad SoftWare Inc., San Diego, CA, USA). The p*K*i values were calculated from the IC_50_ values in accordance with the Cheng–Prusoff equation [55]. The p*K*i values are the mean of at least three independent determinations performed in duplicate.

To define the functional activity of the melatonin analogues at MT_1_ and MT_2_ receptor subtypes, [^35^S]GTPγS binding assays in NIH3T3 cells expressing human-cloned MT_1_ or MT_2_ receptors were performed. The amount of bound [^35^S]GTPγS is proportional to the level of the analogue-induced G-protein activation and is related to the intrinsic activity of the compound under study. The detailed description and validation of this method were reported elsewhere [51, 56]. Membranes (15–25 μg of protein, final incubation volume 100 μL) were incubated at 30°C for 30 min in the presence and in the absence of melatonin analogues in an assay buffer consisting of [^35^S]GTPγS (0.3–0.5 nM), GDP (50 μM), NaCl (100 mM), and MgCl_2_ (3 mM). Nonspecific binding was defined using [^35^S]GTPγS (10 μM). In cell lines expressing human MT_1_ or MT_2_ receptors, melatonin produced a concentration dependent stimulation of basal [^35^S]GTPγS binding with a maximal stimulation, above basal levels, of 370% and 250% in MT_1_ and MT_2_ receptors, respectively. Basal stimulation is the amount of [^35^S]GTPγS specifically bound in the absence of compounds, and it was taken as 100%. The maximal G-protein activation was measured in each experiment by using melatonin (100 nM). Compounds were added at three different concentrations (one concentration was equivalent to 100 nM melatonin, a second one 10 times smaller, and a third one 10 times larger), and the percent stimulation above basal was determined. The equivalent concentration was estimated on the basis of the ratio of the affinity of the test compound to that of melatonin. It was assumed that at the equivalent concentration the test compound occupies the same number of receptors as 100 nM melatonin. All of the measurements were performed in triplicate. The relative intrinsic activity (IAr) values were obtained by dividing the maximum ligand-induced stimulation of [^35^S]GTPγS binding by that of melatonin as measured in the same experiment. By convention, the natural ligand melatonin has an efficacy (*E*_max_) of 100%. Full agonists stimulate [^35^S]GTPγS binding with a maximum efficacy, close to that of melatonin itself. If *E*_max_ is between 30% and 70% that of melatonin (0.3 < IAr < 0.7), the compound is considered a partial agonist, whereas if *E*_max_ is lower than 30% (IAr < 0.3), the compound is considered an antagonist [57].

### Cell culture and reagents

Human MT_1_ and MT_2_ receptors were stably transfected into NIH3T3 mouse fibroblast cells as previously described [52, 53]. Briefly, full-length cDNAs coding for melatonin receptors, cloned from human cerebellum [51], were subcloned into pcDNA INeo (Invitrogen, San Diego, CA, USA) and used to transfect NIH3T3 mouse fibroblast cells by using liposomal transfection kit DOTAP (Boehringer Mannheim, New York, NY, USA), according to the manufacturer's instructions. Selection with G418 (1 mg/ml) started 48 hours after transfection. Stably transfected NIH3T3 cells expressing human cloned MT_1_ (NIH3T3-1A) or MT_2_ (NIH3T3-1B) were cultured in Dulbecco's modified Eagle's medium (DMEM) (Euroclone, Milan, Italy) containing high glucose, 10% bovine calf serum, 1 mM sodium pyruvate and 1 mg /ml G418. Human breast cancer cell lines MCF-7 and MDA-MB231, obtained from American Type Culture Collection (Manassas, VA, USA) were propagated in RPMI 1640 medium (Euroclone, Milan, Italy), supplemented with 10% fetal bovine serum (Opticlone, Euroclone, Milan, Italy), 2 mM L-Glutamine and 100 U/100 μg/ml and Penicillin/Streptomycin. Human melanoma DX3 cells, obtained from dr. A.P. Albino (Memorial Sloan Kettering Cancer Center, New York, NY, USA), and WM-115 cells, obtained from American Type Culture Collection (Manassas, VA, USA), were cultured in DMEM high glucose, supplemented with 10% of fetal bovine serum, 2 mM L-Glutamine and 100 U/100 μg/ml of Penicillin/Streptomycin. All cells were incubated at 37°C with 5% CO2 humidified atmosphere. Melatonin was purchased from Sigma-Aldrich (Milan, Italy).

### Cellular proliferation and viability assay

MCF-7, MDA-MB231, WM-115 and DX3 cells were seeded in 96-well plates at 5.5 × 10^3^, 3 × 10^3^, 7 × 10^3^, 5 × 10^3^ cells/well, respectively and incubated at 37°C with 5% CO_2_ humidified atmosphere. 24 hours later, cells were treated with 0.1% DMSO dissolved in culture medium or with different doses of melatonin, UCM 976, UCM 1032, UCM 1033 and UCM 1037 diluted in 0.1% DMSO and cultured for 24, 48 and 72 hours.

The cell viability and proliferation were assayed using the XTT Cell Viability Assay Kit (Cell Signaling, Euroclone, Milan, Italy), according to the manufacturer's protocol. Briefly, cells were incubated for three hours with freshly prepared XTT solution (50 μL/well) and then the number of viable cells was assessed by measuring the absorbance at 450 nm. The experiments were performed in quadruplicate and repeated three times.

### Apoptosis assay

DX3, WM-115, MCF-7 and MDA-MB231 cells were seeded in 60-mm plates and incubated at 37°C with 5% CO_2_ humidified atmosphere. 24 hours later, cells were treated with 0.1% DMSO dissolved in culture medium or with 10^−4^ M UCM 1037 diluted in 0.1% DMSO. After 24, 48 and 72 hours cells were simultaneously stained with Alexa Fluor 488-conjugated Annexin-V and PI, using the Vybrant Apoptosis Assay kit #2 (Molecular Probes, USA), according to the manufacturer's instructions. Samples were analyzed by FACScalibur flow cytometer (Becton Dickinson Biosciences, San Jose, CA, USA). In each analysis 10,000 events were recorded and the percentage of apoptotic cells estimated by means of the CellQuest Pro software (Becton Dickinson). The simultaneous staining of cells with Annexin-V and Propidium Iodide (PI) allowed the resolution of viable cells (A−/PI−), early apoptotic cells (A+/PI−), necrotic cells (A−/PI+) and late apoptotic cells (A+/PI+).

### Animal experiments

Eight-week-old Swiss male nude mice weighing 22–24 g were purchased from Charles River Laboratory (Calco, Italy). All procedures involving mouse care were in compliance with international directives (directive 2010/63/EU of the European parliament and council; Guide for the Care and Use of Laboratory Animals, United States National Research Council, 2011) and the experimental protocols were authorized by the Committee on Ethics in Animal Experiments of the Italian Minister of Health. Mice were fed a normal mouse diet *ad libitum* and were housed under biosafety level 2 conditions. Experiments were performed under barrier conditions, and sentinel mice were monitored by a quality assurance program.

In each experiment 24 nude mice were injected subcutaneously (s.c.) into the right flank with 1 × 10^6^ human DX3 melanoma cells/mouse. The tumors were allowed to grow for 7 days and when the tumors were detectable, animals were randomly divided into 4 groups (6 mice/group) and treated (s.c. administration) every day with 5% DMSO (control group), UCM 1037, UCM 1033 and melatonin, used at the dose of 16 mg /Kg diluted in 5% DMSO. After 4 weeks from cell injection, all animals were sacrificed and tumors removed and weighted. Experiments were completed three times with similar results.

### Western blot analysis

3 × 10^5^ DX3, WM-115, MCF-7 and MDA-MB231 cells were seeded in 60-mm plates and incubated at 37°C with 5% CO_2_ humidified atmosphere. 24 hours later, cells were treated with 0.1% DMSO dissolved in culture medium or with 10^−4^ M UCM 1037 diluted in 0.1% DMSO and cultured for 10, 30, 60, 120, 240 minutes. Cells were collected by centrifugation at 1000 rpm for 10 min, washed with cold PBS, resuspended in lysis buffer (50 mM Hepes-NaOH, pH 7.5, 150 mM NaCl, 15 mM MgCl_2_, 1 mM EGTA-NaOH pH7.5, 1% Triton X-100, 1 mM sodium orthovanadate, 1 mM phenylmethylsulfonyl fluoride, and 10 μg/ml of leupeptin, aprotinin, antipain, and chymostatin) and incubated on ice for 45 min. The lysates were centrifuged at 13,000 rpm for 10 min at 4°C. Equivalent amounts of proteins were analyzed by SDS–polyacrylamide gel electrophoresis. After electrophoretic separation, the proteins were transferred onto nitrocellulose membrane (GE Healthcare, Pittsburg, PA, USA). After 1 hr of incubation in blocking solution (5% milk in PBS), filters were incubated with the appropriate antibodies: Mel-1A/B-R, Bcl-2 (Santa Cruz Biotechnology, Dallas, TX, USA), Ser473 phosphorylated Akt (p-Akt), Akt, Thr202/Tyr204 phosphorylated p44/p42 MAPK (p-MAPK), MAPK, caspase 3 (Cell Signaling Technology, MA, USA) and α-Tubulin (Sigma-Aldrich). Proteins were visualized with peroxidase-coupled secondary antibody (GE Healthcare), using enhanced chemiluminescence (ECL) for detection (GE Healthcare). Densitometry was performed on scanned immunoblot images using the NIH ImageJ software.

### Statistical analysis

All results were expressed as mean ± standard deviation (s.d.). The significance of differences was evaluated with ANOVA and Bonferroni's test. A probability level of *P* <0.05 was considered statistically significant.

## SUPPLEMENTARY FIGURES



## Abbreviations

MT_1_: melatonin receptor 1
MT_2_: melatonin receptor 2
CREB: cAMP response element-binding protein
MAPK1/2: mitogen-activated protein kinase 1/2
ERK1/2: extracellular signal–regulated kinase 1/2
PLC: phospholipase C
PKC: protein kinase C
PI3K: phosphatidylinositol 3 kinase
DMSO: dimethyl sulfoxide
[^35^S]GTPγS: [^35^S]guanosine-5′-O-(3-thio-triphosphate)
IAr: relative intrinsic activity
PI: Propidium Iodide
p-Akt: Ser473 phosphorylated Akt
p-MAPK: Thr202/Tyr204 phosphorylated p44/p42 MAPK
ANOVA: analysis of variance
s.d.: standard deviation
MLT: melatonin
